# Can Well-Being, Positive Affect, or Contact with the Elderly Be Potential Predictors of Attitudes towards Older People? A Study on the Polish Population

**DOI:** 10.1155/2022/9198970

**Published:** 2022-11-18

**Authors:** Podhorecka Marta, Husejko Jakub, Pyszora Anna, Kędziora-Kornatowska Kornelia, Woźniewicz Agnieszka

**Affiliations:** ^1^Faculty of Health Sciences, Department of Geriatrics, Collegium Medicum in Bydgoszcz, Nicolaus Copernicus University in Toruń, Poland; ^2^Faculty of Health Sciences, Department of Palliative Care, Collegium Medicum in Bydgoszcz, Nicolaus Copernicus University in Toruń, Poland

## Abstract

**Objectives:**

The age discrimination, i.e., ageism, is still a current social problem. Therefore, it is justified to conduct studies increasing the knowledge about this phenomenon. The aim of our research was to determine whether the type of personality, manifested mood, and well-being can influence the attitudes towards the elderly. *Material and Methods*. During the research, we collected information from 923 participants and we used the following tools: demographic questionnaire, Kogan's Attitudes Toward Old People Scale, Euthymia Scale, WHO-5 Well-Being Index, and the author's questionnaire on contacts with an elderly person.

**Results:**

We used R 4.0.2 to analyse the data. In our current model study, we did not observe statistically significant relationships between the WHO-5 or ES scores and the KOAP score.

**Conclusions:**

The conducted study did not show any correlation between mood, sense of well-being, or contact with the elderly and attitude towards the elderly. The results of our study may become the basis for further research to find the relationship between the mood and well-being shown in attitudes towards the elderly. Perhaps, however, the assumption should also be made that there is no such relationship.

## 1. Introduction

Compared to other described processes, which boil down to the exclusion of specific social groups, such as sexism or racism, ageism has been noticed and described relatively recently [1]. The current definition, developed by Iversen et al. in 2009, can be characterized as “negative or positive stereotypes, prejudices and/or discrimination (or an advantage) against people based on their chronological age. Ageism can be hidden or explicit, and it can be expressed at the micro, meso or macro level” [2]. The latest research on the phenomenon of ageism in individual age groups has shown that the phenomenon of discrimination is more often noticed and reported by young people, but this process is common in all groups at risk of exclusion on the basis of age [3].

The influence of mood and self-feeling on the phenomenon of stereotyping, which is the main factor that may lead to the development of ageism, has already been described many times. In a study conducted almost 30 years ago, in which the respondents were evoked positive, neutral, and negative moods, a different perception of minority social groups in the context of their stereotyping was noticed [4]. These observations were corroborated in another study, which also induced a certain mood in participants, thanks to which it was noted that in people with a negative mood and malaise, the stereotyping process may be more radical [5].

When trying to determine the influence of both mood and well-being on the tendency to age discrimination, one should not forget about the influence of time spent in the company of elderly people, which may also be important in shaping attitudes towards older people [6]. Based on the research conducted so far on the phenomenon of exclusion of the elderly, we have put forward a hypothesis that the above-mentioned factors may be potential predictors of attitudes towards the elderly in Polish society.

## 2. Material and Methods

### 2.1. Objectives

The aim of our research was to determine whether the type of personality, manifested mood, and well-being can influence attitudes towards the elderly. We also asked detailed research questions:

- Can attitudes towards older people be associated with our positive affect?
- Can attitudes towards older people be associated with our well-being?
- Can attitudes towards older people be associated with contact with the elderly?

### 2.2. Participants

The study was conducted on Polish society. Participation was voluntary and anonymous. It was a cross-sectional online survey conducted in February 2021 using the Survgo system. The population of Poland is estimated at around 38,265,000. 923 people took part in our study, which is a representative group, but due to the form of the project, we cannot treat it as such.

When completing the database, we wanted the distribution in individual age groups and gender distribution to be proportional. Only fully completed adult questionnaires were included in the analysis.

### 2.3. Methods

During the research, we used the following tools: demographic questionnaire, Kogan's Attitudes Toward Old People Scale, Euthymia Scale, and WHO-5 Well-Being Index. Kogan's Attitudes Toward Old People Scale (KAOP) contains 34 statements which the respondent chooses from 6-point Likert answers (1-strongly disagree and 6-strongly agree) [7]. The respondent could receive from 34 to 204 points. Higher scores indicate a more positive attitude towards older people, and lower scores indicate a more negative attitude towards the elderly [8].

We used the 10-item Euthymia Scale (ES) [9] to assess the manifested mood. Each question of the questionnaire could be marked either true or false. The presented tool was based on Jahoda's conceptualization of euthymia [10, 11].

Another tool used was the WHO-5 index, which we used to assess well-being, applying a 6-point Likert-like scale (0, “at no time,” to 5, “all the time”). The maximum number of points was 100, and scores < 50 suggesting impaired well-being were assumed, while ≤28 indicate likely depression [12].

The last used tool was the proprietary questionnaire with questions about one's own experiences in the field of contacts with the elderly (Table 1).

### 2.4. Ethical Approval

The study was approved by the Bioethics Committee of the Nicolaus Copernicus University Collegium Medicum in Bydgoszcz, Poland (KB 83/2021). The research was conducted in accordance with the Helsinki Declaration. All participants provided informed consent for the research.

### 2.5. Data Analysis

We used R 4.0.2 to analyse the data [13]. To model the KOAP score as a function of the predictors, we used Bayesian robust linear regression with *t* distribution [14]. In each of the analyses, the “no opinion” response was assumed to be equivalent to neutral attitude and constituted a midpoint of the scale. Ordered categorical predictors were coded with orthogonal linear contrast, unordered categorical predictors were coded with sum-to-zero contrast, and continuous predictors were entered into a model on a standardized scale.

In Bayesian statistics, the inference is based on analysing the posterior probability distributions of a model parameters (e.g., regression weights), obtained by integrating likelihood (data) with prior probability distributions. Regression weight is said to be statistically credible when 95% credible intervals (95% CI) of the posterior distribution exclude zero [14]. A point estimate of the effect means the posterior distributions are presented. Default improper flat priors were used for the regression weights.

To investigate the relationship between dependent variables, credible predicted marginal means with corresponding 95% CI are presented in figures. These values represent the median of a posterior distribution of the predicted KOAP values.

To approximate posterior distributions of the models, Markov chain Monte Carlo (MCMC) sampling procedure was used via brms package [15]. Six parallel chains were used, each consisting of 8,000 samples, with 4,000 samples used as warm-up period and every 10th sample recorded, resulting in 2,400 recorded samples in total. Sampling procedure was efficient and resulted with well-mixed and not autocorrelated chains and unimodal posteriors. Model accuracy was assessed with posterior predictive checks [16].

## 3. Results

The characteristics of the participants are presented in Table 2, and descriptive statistics for KOAP, WHO-5, and ES are presented in Table 3.

Model coefficients of the Bayesian robust linear regression with KOAP as dependent variable, WHO-5 and ES scores as predictors, and frequency of contacts with the elderly with professional status as additional control variables (these variables were shown to correlate with KOAP in an investigation reported elsewhere [17]) are summarized in Table 4, and the model predictions are presented in Figure 1. We did not observe statistically credible relationships between WHO-5 or ES scores and the KOAP score in the tested model.

## 4. Discussion

The most important findings of our study were that the levels of well-being and euthymia in the participants of our study were low.

Recognizing low levels of well-being is clinically important, because it affects the overall functioning of the patient and may affect the manifestation of symptoms, their severity, or the patient's concentration on negative aspects. It should be noted that the tools we used (WHO-5 Well-Being Index [12] and Euthymia Scale [9]) contain positively formulated statements, in contrast to other scales focusing on negative symptoms or problems reported by the evaluated persons [18, 19]. Considering the low result obtained in our own research, it is worth screening the level of well-being in order to struggle with people at risk of mental difficulties in the future, or those already struggling with them and not covered by appropriate medical care, and if appropriate, proposing professional support.

It is possible that the low result was influenced by the period of time in which the research was conducted, namely, the period of the COVID-19 pandemic. It is worth emphasizing the relatively low average point value in the WHO-5 Well-Being Index obtained by the participants of the study. It amounted to 54.87 points, where the value < 50 suggests poor emotional well-being and is a sign for further testing [12]. The impact of the duration of the study during the SARS-CoV-2 pandemic on the results obtained is corroborated by the results of studies conducted by White and Van Der Boor among 600 British, where the mean WHO-5 point value was 41.72. The authors of the study emphasize that both self-isolation before official closure and the feeling of isolation during a pandemic were associated with poorer mental health, general well-being, and quality of life [20]. Our participants' results are lower (for both WHO-5 and ES) than the average reported in another study that was also conducted online also during the pandemic period [21].

In our study, we did not observe statistically significant relationships between the sense of well-being assessed in the WHO-5 Well-Being Index scale and ageism, nor statistically credible relationships between Euthymia Scale results and ageism. However, there are some critical points to be made with regard to our research methodology itself; for example, some people with a specific personality are involved in filling out questionnaires at all [22]. Despite the possible limitations, the study has many strengths—a large research sample and multifaceted approach to the phenomena of ageism contribute to deepening the knowledge in this field.

Research on personality and manifested attitudes towards the elderly was also undertaken by Allan et al., who observed a relationship with attitudes towards old age, where personality traits (except extraversion) had a direct or indirect impact on attitudes towards the elderly [23]. In other studies, the authors also emphasize the relationship between the fear of death and dying and ageism, where it was corroborated that agreeableness, openness, and fear of death of others were negatively related to the phenomenon of ageism [24].

## 5. Limitation

We did not observe statistically significant relationships between the sense of well-being assessed in the WHO-5 Well-Being Index scale and ageism, nor statistically credible relationships between Euthymia Scale results and ageism. Both self-isolation before official closure and the feeling of isolation as well as concerns about the continuing pandemic were associated with poorer mental health, general well-being, and quality of life [20]. Unfortunately, the study itself showed many limitations in the research tool used to assess personality. It can be assumed that active Internet users or people who voluntarily and willingly participate in the survey may also represent certain personality types [25–27]. In the future, it would be useful to take advantage of the marked expansion of the literature and to consider the choice of this instrument and also to develop methodologies for individual meetings with respondents.

## 6. Conclusion

The conducted study did not show any correlation between mood, sense of well-being, or contact with the elderly and attitude towards the elderly. The results of our study may become the basis for further research to find the relationship between the mood and well-being shown in attitudes towards the elderly. Perhaps, however, the assumption should also be made that there is no such relationship. Regardless of the position taken, research in this area should be continued, as it will allow the development of measures to reduce ageism. Future studies may consider the potential role of a pandemic or include postpandemic data collection.

## Figures and Tables

**Figure 1:** Posterior medians (black points and blue line) of the predicted mean KOAP scores as a function of tested predictors (including MBTI not shown in Table 3). Vertical lines and shaded area are 95% credible intervals. Note: KOAP, WHO-5, and ES are on a standardized scale. Grey transparent points show data.

**Table 1:** The original questionnaire “contact with the elderly”.

Contact with the elderly		
1	Do you live or have you ever lived with an elderly person?	(a) Yes (b) No

2	Do you have contact with the elderly in your private life?	(a) Yes, I live with an elderly person (b) Yes, several times a week (c) Only at ceremonies (d) Occasional (e) Not at all

3	Do you have contact with people over 65 at work?	(a) Yes (b) No (c) I do not have the opportunity

4	Are you in contact with elderly people who are not family members?	(a) Yes (b) No (c) I do not have the opportunity

5	How important are contacts with the elderly to you?	(a) Very important (b) Important (c) It does not matter (d) They are not important

**Table 2:** Characteristics of participants (*n* = 923).

	Freq	Prop
*Gender*		
Female	475	51.46
Male	448	48.54
*Age*		
18-29	251	27.19
30-39	233	25.24
40-49	234	25.35
≥50	205	22.21
*Place of residence*		
Village	163	17.66
<50 K	207	22.43
<100 K	159	17.23
<250 K	138	14.95
>250 K	256	27.74
*Marital status*		
Single	158	17.12
Informal relationship	225	24.38
Married	482	52.22
S/D/W	58	6.28
*Education*		
Elementary	28	3.03
Vocational	98	10.62
Secondary	407	44.1
Higher	390	42.25
*Professional situation*		
At school	73	7.91
Unemployed	81	8.78
Employed	686	74.32
Pensioner	83	8.99
*Annual income*		
0–20.999	153	16.58
21.000–40.999	220	23.84
41.000–60.999	215	23.29
61.000–80.999	151	16.36
81.000 and more	117	12.68
Refuse to answer	67	7.26

**Table 3:** Descriptive statistics.

	M	SD	Min	Q_1_	Me	Q_3_	Max
KOAP	90.88	17.41	0	83	89	101	170
WHO-5	54.87	20.86	0	40	56	68	100
ES	2.77	2.58	0	1	2	4	10

Note: M: mean; SD: standard deviation; Min: minimum; Q_1_: first quartile; Me: median (second quartile); Q_3_: third quartile; Max: maximum.

**Table 4:** Results of Bayesian robust linear regression with KOAP score as dependent variable.

	*β*	SE	LI	UI
Intercept	-0.19	0.05	-0.28	-0.1
Marital status (single)	-0.19	0.07	-0.33	-0.04
Marital status (informal relationship)	0.17	0.07	0.04	0.32
Marital status (married)	-0.1	0.04	-0.19	-0.02
Frequency of contacts with the elderly	0.96	0.09	0.78	1.13
WHO-5	0.03	0.03	-0.04	0.09
ES	-0.04	0.03	-0.1	0.03
*σ*	0.65	0.03	0.6	0.71
*ν*	5.11	0.92	3.68	7.28
Bayesian *R*^2^	0.25	0.02	0.21	0.29

Note: *β* and SE are posterior mean and standard error of the mean, respectively. LI and UI are lower and upper boundaries of the 95% credibility interval. Parameters *σ* and *ν* are the scale and normality parameters of the *t* distribution, respectively.

## Data Availability

Data are available on request from the corresponding author marta.podhorecka@cm.umk.pl).
